# Emotion Analysis Model of Microblog Comment Text Based on CNN-BiLSTM

This article has been retracted.

**DOI:** 10.1155/2022/1669569

**Published:** 2022-04-30

**Authors:** Aichuan Li, Shujuan Yi

**Affiliations:** ^1^College of Information and Electrical Engineering, Heilongjiang Bayi Agricultural University, Daqing, Heilongjiang 163319, China; ^2^Engineering Research Center of Processing and Utilization of Grain By-Products, Ministry of Education, Heilongjiang Engineering Technology Research Center for Rice Ecological Seedlings Device and Whole Process Mechanization, Daqing, Heilongjiang 163319, China

## Abstract

Aiming at the problems of over reliance on labor and low generalization of traditional emotion analysis methods based on dictionary and machine learning, an emotion analysis model of microblog comment text based on deep learning is proposed. Firstly, text is obtained through microblog crawler program. After data preprocessing, including data cleaning, Chinese word segmentation, removal of stop words, and so on, the Skip-gram model is used for word vector training on a large-scale unmarked corpus, and then the trained word vector is used as the text input of CNN-BiLSTM model, which combines Bidirectional Long-Short Term Memory (BiLSTM) neural network and Convolution Neural Network (CNN). Considering the historical context information and the subsequent context information, BiLSTM can better use the temporal relationship of text to learn sentence semantics. CNN can extract hidden features from the text and combine them. Finally, after Adamax optimization training, the emotion type of microblog comment text is output. The proposed model combines the learning advantages of BiLSTM and CNN. The overall accuracy of text emotion analysis has been greatly improved, with an accuracy of 0.94 and an improvement of 8.51% compared with the single CNN model.

## 1. Introduction

With the rapid development of information technology and the growing number of Internet users, the Internet has been inseparable from people's daily life and information has begun to show explosive growth [1]. Microblog is one of the main public opinion platforms in China, carrying a large number of information released by the public. Most of these information have emotional tendencies [2, 3]. Analyzing the text of microblog hot topics and mining the emotional tendencies are of great significance for government units or enterprises to understand the trend of public opinion [4].

Text emotion analysis refers to the analysis of subjective text with emotional color, mining the contained emotional tendency, and dividing the emotional attitude [5]. Microblog text emotion analysis belongs to a specific research field of text emotion classification. In the research field of natural language processing, the analysis and research of text emotion is an important branch. The process of text emotion analysis includes the acquisition of original data, data preprocessing, feature extraction, classifier, and emotion category output [6–8]. The acquisition of original data is generally through web crawlers to obtain relevant data; data preprocessing refers to data cleaning to remove noise. Common methods include removing invalid characters and data, unifying data categories, using word segmentation tools for word segmentation, stop word filtering, etc. Feature extraction has different implementation methods according to the different methods used, and the feature extraction of deep learning method is generally automatic [9]. The final emotional category of the text is obtained from the output of the classifier. The common classifiers are Support Vector Machine and Softmax.

In foreign countries, many achievements have been made in the emotional analysis of Twitter texts. However, in China, the research on Chinese text begins relatively late, and the research on Chinese microblog text is relatively few. Due to the differences of language expression and the diversity and complexity of Chinese expression, the research on microblog text is full of challenges [10, 11]. Reference [12] analyzed and expounded the level of emotion analysis, various emotion models, emotion analysis, and text emotion detection process, and discussed the challenges faced in the process of emotion analysis. Reference [13] proposed a dictionary-based text emotion analysis system. This method is the main standard method for modeling text for machine learning in emotion analysis methods, which can effectively solve the problem of data overload. But the method is more traditional and difficult to apply to the complex text environment of microblog. Reference [14] developed a classification model based on machine learning algorithm to realize the social website automatically filtering out the messages from the visitors for avoiding excessive speech, but the performance of the single model was slightly deficient. The traditional model based on motion dictionary is simple, fast, and stable, but it also has limitations. The traditional model needs to prepare a relatively complete motion dictionary, but this step needs a lot of human and material resources for careful operation, which has low practicability and is not conducive to the development of natural language processing.

With the continuous development of machine learning, some inherent advantages of deep learning have solved some problems. Deep learning can establish a classification model for the emotion classification of microblog text without background language knowledge to realize the emotion classification of microblog text with high accuracy [15]. For example, reference [16] proposed an image text emotion analysis model based on deep multimodal attention fusion, which used the hybrid fusion framework for emotion analysis, and realized emotion classification and recognition by combining the discriminant features and internal correlation between visual and semantic content. Reference [17] proposed a Chinese text emotion analysis method based on Convolutional Neural Network (CNN), which realized feature preprocessing by normalizing features, and optimized text feature size to improve analysis performance. However, the CNN model ignores the correlation between the whole and the part, and the analysis accuracy of comment text needs to be further improved. Reference [18] proposed a network text emotion analysis method based on the improved attention mechanism and two-way gated loop unit model. Reference [19] proposed a text emotion analysis method combining dictionary language model and deep learning to solve the problem of accurate and rapid emotion analysis of comment text in the network big data environment.

Aiming at the problems of single word quantization and poor analysis accuracy in most of the existing deep learning algorithms in text processing, an emotion analysis model of microblog comment text based on deep learning is proposed. Compared with the traditional dictionary-based and machine learning models, the innovations of the proposed model are as follows.

1. In order to better analyze emotion, the Skip-gram model is used to quantify the word of the preprocessed text data set. Part of the speech features are integrated, which can significantly improve the effect of emotion analysis.
2. Because the output of LSTM hidden layer only depends on the output of the previous time, resulting in inaccurate analysis results, the proposed model combines Bidirectional Long Short-Term Memory (BiLSTM) and CNN to construct CNN-BiLSTM model. BiLSTM can obtain previous and subsequent information, and CNN can deeply mine text features. Thus, the accuracy of text emotion analysis is improved.

## 2. Proposed Model

### 2.1. Model Process

The process of microblog comment text emotion analysis model based on deep learning is shown in Figure 1, which mainly includes four parts: text data acquisition, text preprocessing, text vectorization, and neural network model.

After the text data is obtained, it is divided into training data set and test data set through manual annotation, and the data set is preprocessed through data cleaning, Chinese word segmentation, and removal of stop words, and then the text vectorization is completed. Finally, the quantified text is sent to CNN-BiLSTM model for emotional analysis of microblog comment text.

#### 2.1.1. Text Acquisition

In order to construct the word vector of words and emoticons, a microblog crawler program is implemented by using the open-source crawler framework WebCollecter, and the crawled microblog text is segmented by using Natural Language Processing and Information Retrieval (NLPIR) tool. In the process of word segmentation, the emotional symbols in the constructed microblog emotional symbol database are used as a word segmentation dictionary to make them exist as a basic language unit after word segmentation [20, 21]. In addition, a series of microblog text preprocessing has been carried out, such as complex and simple conversion, replacement of Uniform Resource Locator (URL), elimination of short and meaningless microblogs, etc. Finally, a Word2Vec word vector training corpus is constructed, including 40302879 microblogs and 1432646813 words. Skip-gram model is used in the training process, and other relevant parameters are set by default. After training, a word vector space containing 850599 words is obtained, in which the word vector dimension of each word is 250.

#### 2.1.2. Text Preprocessing

Generally, the obtained text data has many invalid contents or dirty data that affect the later classification, so text preprocessing is an essential work, and good text preprocessing can improve the accuracy of later classification [22]. Text preprocessing generally includes three steps: data cleaning, Chinese word segmentation, and removing stop words.

*(1) Data Cleaning*. Data cleaning is to clean and remove characters and data irrelevant to text content. Taking the microblog text as an example, there are some irrelevant characters and data in the microblog text, such as forwarding symbol //, designated user symbol @, topic symbol #, microblog expression, HTML tag, URL link, and so on, which are irrelevant to the content expressed by the microblog and can affect the result of emotion analysis task. For these data, the strategy of deletion or replacement can be adopted. The regular expression is used to delete the character data other than the microblog expression, and the microblog expression is replaced with the corresponding Chinese text.

*(2) Chinese Word Segmentation*. Because Chinese text is not like English text, which is naturally separated by spaces, word segmentation must be done for Chinese text, and a Chinese text must be divided into individual words. At present, Chinese word segmentation can be divided into two methods: machine learning-based and rule-based (rule refers to word segmentation specification and thesaurus). In 2002, researchers treated Chinese word segmentation as part of speech tagging. After tagging each word, they used a supervised machine learning model for word segmentation. Then, the fusion model of BiLSTM and Conditional Random Field (CRF) was used for Chinese word segmentation. At the same time, the research showed that the machine learning method based on statistics was better than the traditional rule-based method, especially in the recognition of unlisted words (words not included in the dictionary). With the development of deep learning, deep learning has begun to be applied in the field of emotion analysis. Although deep learning has not shown excellent technical advantages over the traditional supervised machine learning method, it still has potential. In the proposed method, word segmentation is only a pre-step in the text emotion analysis task, so it is decided to use the existing Jieba Chinese word segmentation tool for word segmentation.

*(3) Remove Stop Words*. Similar to information retrieval, in which some words shielded in order to improve query efficiency and save storage space, in the text emotion analysis task, some words unrelated to emotional tendency will also be removed, which are called stopwords. In Chinese text, in addition to nouns, adjectives, verbs, adverbs, and other emotional words, there are also some meaningless words, such as “do, bar, do, also, to, from, then, in addition, then”. These meaningless words generally belong to prepositions, mood auxiliaries, and conjunctions. Removing these meaningless stopwords through the stopwords list can reduce the dimension of feature vector and reduce data noise and data volume.

#### 2.1.3. Text Vectorization

The word sequence obtained through text preprocessing needs to be transformed into a vector used as the final input of the model [23]. Word2Vec launched by Google is a commonly used word vector tool, which is mainly based on Continuous Bags of Words (CBOW) model and Skip-gram model. The structures of the two models are shown in Figure 2. CBOW model uses the context of the current word *c*_*t*_ to predict the probability of the current word *c*_*t*_, and Skip-gram model uses *c*_*t*_ to predict the probability of its context. The proposed model uses Skip-gram model to train word vectors on large-scale unmarked corpus, and takes the trained word vectors as the input word vectors of the model.

Skip-gram neural network model can be constructed and implemented through two frameworks: Hierarchical Softmax and Negative Sampling (NEG). The proposed model adopts the method of Negative Sampling, including three-layer structure of input layer, projection layer, and output layer. The text samples *c*_*t*−*n*_,…, *c*_*t*−1_, *c*_*t*_, *c*_*t*+1_,…, *c*_*t*+*n*_ in Corpus are recorded as samples (*c*, context(*c*)). The Negative Sampling method divides words into positive samples and negative samples. The central word *c* is negative samples, and the rest are positive samples. In the output layer, the Negative Sampling technology is adopted. For any *ϖ* ∈ {*u*} ∪ NEG(*u*), NEG(*u*) represents negative sample set generated when processing word *u*, the posterior probability of which is as follows:

(1) $$\begin{array}{c} p\left(\varpi |c\right)=\left\{\begin{array}{c} \sigma \left(v{\left(c\right)}^{T}\theta^{\varpi }\right),L^{u}\left(\varpi \right)=1,\\ 1-\sigma \left(v{\left(c\right)}^{T}\theta^{\varpi }\right),L^{u}\left(\varpi \right)=0, \end{array}\right. \end{array}$$

where *σ* represents Sigmoid activation function; *v*(*c*) represents the target word; and *θ* represents the *ϖ*-th word in the window except the target word.

The Skip-gram language model requires to maximize the probability of words appearing in the context. The optimized objective function is in the following form:

(2) $$\begin{array}{c} G=\prod_{c\in C}\prod_{u\in \text{Context}\left(c\right)}\prod_{\varpi \in \left\{u\right\}\cup \text{NEG}\left(u\right)}p\left(\varpi |c\right),\\ L=\sum_{c\in C}\sum_{u\in C\left(c\right)}\sum_{\varpi \in \left\{u\right\}\cup \text{NEG}\left(u\right)}\begin{array}{c} \left\{L^{u}\left(\varpi \right)\cdot \log\left[\sigma \left(v{\left(c\right)}^{T}\theta^{\varpi }\right)\right]\right\}+\\ \left[1-L^{u}\left(\varpi \right)\right]\cdot \log\left[\sigma \left(v{\left(c\right)}^{T}\theta^{\varpi }\right)\right] \end{array}. \end{array}$$

### 2.2. Text Emotion Analysis Based on CNN-BiLSTM

#### 2.2.1. CNN-BiLSTM Model Structure

The hidden layer output of the standard LSTM at a certain time only depends on the output of the previous step, so it is only related to the pre-context, that is, it can only see the historical information. However, in the actual situation of text emotion analysis, it should be related to both the pre-context and the post-context, that is, it can not only see the historical information, but also pay attention to the future information [24]. BiLSTM can exactly do this because it can obtain both positive and reverse semantic information. Its model structure is shown in Figure 3.

Therefore, the proposed model uses the fusion of BiLSTM and CNN to construct the CNN-BiLSTM model, and its structure is shown in Figure 4. The input of the model is the word vector matrix integrating part of speech features trained by Word2Vec tool, and the output is the text emotion classification result.

#### 2.2.2. Convolution

The convolution layer uses convolution kernel to perform convolution abstract operation on text word vector, so that the original word vector sequence becomes a convoluted abstract meaning sequence. For a given text sample **x**, it can be expressed as **x**=(**x**_1_, **x**_2_,…, **x**_*n*_), where **x**_*i*_ ∈ **R**^*d*^ represents the *d* dimension word vector of the *i*-th word in the text sample **x**. *n* represents the number of words in the text, so the text sample can be expressed as **x** ∈ **R**^*n*×*d*^. The number of words contained in the convolution kernel is *k*, and its vector is **m** ∈ **R**^*k*×*d*^. Usually in image processing, the convolution kernel is square, such as 6 × 6. Then, the convolution operation is performed by gradually moving the convolution kernel along the width and height on the picture. However, since the input in the natural language processing task is a *n* × *d* dimensional word matrix, the convolution kernel slides only in height, but in width, it is consistent with the dimension of the word vector [25]. This ensures that the position of each window sliding is a complete word vector without convolution of some word vectors of several words, and ensures the rationality of words as the minimum granularity in the language. Therefore, for each position *i* in the text sample **x**, there is a window vector **s**_*i*_ containing a continuous *k* word vectors, which is expressed as follows:

(3) $$\begin{array}{c} s_{i}=\left[x_{i},x_{i+1},\ldots ,x_{i+k+1}\right]. \end{array}$$

The feature map *φ* ∈ **R**^*n*−*k*+1^ is calculated by sliding the windows one by one through the convolution kernel, *φ*=[*φ*_1_, *φ*_2_,…, *φ*_*n*−*k*+1_]. The calculation of *φ*_*i*_ in each sliding window is as follows:

(4) $$\begin{array}{c} \varphi_{i}=\delta \left(\omega_{i}*m+b\right), \end{array}$$

where *∗* represents the multiplication of corresponding matrix elements, **b** is the offset vector, function *δ* is the activation function, and *ω* is the weight matrix. The proposed model selects ReLU function as the activation function.

The designed convolution layer generates multiple feature maps through *j* convolution kernels, and all convolution kernels have the same size. *j* feature maps are obtained from the window vector **s**_*i*_ at each position *i* in the text sample **x**, and a new feature representation Ψ_*i*_ is obtained by combining the feature vectors *φ*_*i*_ at the same position:

(5) $$\begin{array}{c} \Psi_{i}=\left[\varphi_{i1},\varphi_{i2},\ldots ,\varphi_{ij}\right]. \end{array}$$

The final feature representation is Ψ ∈ **R**^(*n* − *k*+1)×*j*^. Ψ=[Ψ_1_, Ψ_2_,…, Ψ_*j*_] is used as the input of the next Max-pooling layer.

#### 2.2.3. Pooling Layer

In the convoluted feature maps, the average pooling or Max pooling is usually used to reduce the amount of data, so as to reduce the parameters and reduce the amount of calculation. The proposed model adopts the Max-pooling method, and the mathematical expression is as follows:

(6) $$\begin{array}{c} \tilde{\varphi }=\max\left(\varphi_{i}\right). \end{array}$$

It can be seen from equation (6) that for the feature maps obtained by convolution kernel, only the feature map with the highest score is retained.

There are two reasons for using the Max-pooling method. First, the calculation of the upper layer is reduced by eliminating the non-maximum value, and the most significant information can be retained by extracting the local dependencies of different convolution kernels.

#### 2.2.4. BiLSTM Layer

The deep features after Max pooling will be used as the input of BiLSTM in this layer. Compared with LSTM, BiLSTM can focus on the future context on the basis of considering the past context. In addition, when accepting text vectors, the order is from left to right, which will lead to the more backward words that are more likely to affect the emotion of the whole sentence, which is unreasonable. BiLSTM can better alleviate this. The hidden layer of BiLSTM includes forward connection and backward connection, which are used to learn the forward information and backward information of text, respectively, and are both connected to the output layer unit. The backward connection output vector is obtained through the following operations:

(7) $$\begin{array}{c} {\overset{\leftarrow }{f}}_{t}=\sigma \left({\overset{\leftarrow }{\omega }}_{1f}x_{t}+{\overset{\leftarrow }{\omega }}_{2f}h_{t+!}+{\overset{\leftarrow }{b}}_{f}\right),\\ {\overset{\leftarrow }{\phi }}_{t}=\sigma \left({\overset{\leftarrow }{\omega }}_{1i}x_{t}+{\overset{\leftarrow }{\omega }}_{2i}h_{t+!}+{\overset{\leftarrow }{b}}_{i}\right),\\ {\overset{\leftarrow }{C}}_{t}={\overset{\leftarrow }{f}}_{t}*{\overset{\leftarrow }{C}}_{t+1}+{\overset{\leftarrow }{\phi }}_{t}*\tanh\left({\overset{\leftarrow }{\omega }}_{1c}x_{t}+{\overset{\leftarrow }{\omega }}_{2c}h_{t+!}+{\overset{\leftarrow }{b}}_{c}\right),\\ {\overset{\leftarrow }{o}}_{t}=\sigma \left({\overset{\leftarrow }{\omega }}_{1o}x_{t}+{\overset{\leftarrow }{\omega }}_{2o}h_{t+!}+{\overset{\leftarrow }{b}}_{o}\right),\\ {\overset{\leftarrow }{h}}_{t}={\overset{\leftarrow }{o}}_{t}*\tanh\left({\overset{\leftarrow }{C}}_{t}\right), \end{array}$$

where ${\overset{\leftarrow }{f}}_{t}1/2$, ${\overset{\leftarrow }{\phi }}_{t}$, ${\overset{\leftarrow }{o}}_{t}$ are the outputs of backward LSTM forgetting gate, input gate and output gate at time *t*, respectively; ${\overset{\leftarrow }{C}}_{t}$ represents the output of the backward memory control unit after time *t*. ${\overset{\leftarrow }{\omega }}_{1}$ and ${\overset{\leftarrow }{\omega }}_{2}$ are the weight matrices of backward categories, and its subscript represents the specific category; **x**_*t*_ and **h**_*t*+1_ represent the input and hidden layer vectors at time *t* and, *t*+1 respectively; $\overset{\leftarrow }{b}$ represents the backward offset vector, and its subscript represents the specific category.

Finally, the output vector representation **h** of BiLSTM hidden layer is the combination of forward connection output $\overset{⟶}{h}$ and backward connection output $\overset{\leftarrow }{h}$, and also serves as the input of the next layer:

(8) $$\begin{array}{c} h=\left[\overset{⟶}{h}⊕\overset{\leftarrow }{h}\right]. \end{array}$$

#### 2.2.5. Full Connection Layer and Classifier

The full connection layer receives the output features of the BiLSTM layer as the input, and then outputs them to the final output layer after comprehensive processing. Each neuron in the full connection layer is connected to all neurons in the previous layer in order to integrate features.

The output layer selects Softmax as the classifier, which outputs the results of text emotion analysis. The Softmax classifier is calculated as follows:

(9) $$\begin{array}{c} p_{i}=\frac{e^{\left(\vartheta_{i}^{T}x\right)}}{\sum_{q=1}^{Q}e^{\left(\vartheta_{q}^{T}x\right)}}, \end{array}$$

where *p*_*i*_ represents the probability that the classification result is category *i*; *Q* indicates the number of all categories; and *ϑ*_*i*_^*T*^*x* represents multiple inputs. Each output is in the interval [0, 1], the probability sum of all categories is 1, and the category with the highest probability is taken as the final result of the text emotion analysis task.

### 2.3. Optimization Algorithm

As everyone knows, the optimization algorithm plays an important role in the success or failure of the deep neural network model. Because the main role of the optimization algorithm is to find the global optimal solution by gradient descent in the back propagation of neurons and update the connection weight of neurons, an excellent optimization algorithm can accurately find the global optimal solution in the shortest time and accurately update the weight matrix of connected neurons. Different optimization algorithms are selected for the same model to produce different results. Common optimization algorithms include Stochastic Gradient Descent (SGD), RMSprop, Adadelta, Adam, etc. The proposed model adopts Adamax optimization algorithm, which is a variant of Adam algorithm. Adam optimization algorithm is a random objective function optimization algorithm based on adaptive estimation of low-order matrix proposed by Diederik P. Kingma et al. in 2015. This method has the advantages of simple implementation, high calculation efficiency, and less memory requirements. It is very suitable to solve the problem of large data and parameter scale.

In Adam, the gradient of each individual weight in the update rule is inversely proportional to the L2 norm of the gradient at the current time and the previous time, so the update rule based on L2 norm can be extended to the update rule based on LP norm. With the increase of *p*, it begins to become numerically unstable. In the special case of *p* ⟶ ∞, the original algorithm becomes a very simple and stable algorithm, which is Adamax. Its description is shown in algorithm 1.

## 3. Experiment and Analysis

The specific parameters of the microblog data set used in the experiment, such as sentence length, batch size, and Dropout value, are shown in Table 1. The server hardware environment used in this experiment is: graphics card GTX1080Ti dual card, 22 G video memory, CPU2.6 GHz, 16 threads, 16 G memory capacity, and 240 G hard disk capacity; and the operating system is Ubuntu 16.04.

### 3.1. Evaluation Criteria

The proposed model uses Precision and Recall as the indicators to evaluate the results of emotion classification in positive emotion samples and negative emotion samples, respectively, and Accuracy is used as the evaluation index for the overall performance. TP (True Positive) represents the number of samples with positive emotion and correctly predicted as positive samples; FP (False Positive) indicates the number of samples with negative emotion and incorrectly predicted as positive samples; TN (True Negative) indicates the number of samples with negative emotion and correctly predicted as negative samples; FN (False Negative) indicates the number of samples with positive emotion and incorrectly predicted as negative samples.

(1) Precision, representing the proportion of text correctly classified into this category in text actually classified into this category, is calculated as follows:
  (10) $$\begin{array}{c} {\text{Precision}}_{p}=\frac{\text{TP}}{\text{TP}+\text{FP}},\\ {\text{Precision}}_{n}=\frac{\text{TN}}{\text{TN}+\text{FN}}. \end{array}$$
(2) Recall, representing the proportion of text correctly classified into this category in all text of this category, is calculated as follows:
  (11) $$\begin{array}{c} {\text{Recall}}_{p}=\frac{\text{TP}}{\text{TP}+\text{FN}},\\ {\text{Recall}}_{n}=\frac{\text{TN}}{\text{TN}+\text{FP}}. \end{array}$$
(3) Accuracy, the proportion of correct prediction, is calculated as follows:

(12) $$\begin{array}{c} \text{Accuracy}=\frac{\text{TP}+\text{TN}}{\text{TP}+\text{TN}+\text{FP}+\text{FN}}. \end{array}$$

### 3.2. Effect of Epoch Parameter on Model Results

In deep learning, Epoch refers to a complete iteration, including a forward transfer and a reverse transfer of all the training samples. The experiment is based on CNN-BiLSTM model. Except for Epoch parameters, other parameters remain unchanged. The accuracy under different Epochs is shown in Figure 5.

As can be seen from Figure 5, with the increase of Epoch, the accuracy of the training set in the text emotion analysis task continues to improve, while the test set first increases and then decreases. When the 7th Epoch is trained, the accuracy on the test set reaches the maximum, and then the accuracy begins to decline, which may be due to over-fitting at the beginning of training. It can be concluded that too much or too little Epoch values have an impact on the results of text emotion analysis. When there is too little Epoch, the optimal results will not be obtained, but when there are too many training times, the model will over fit the training data and perform poorly in the test set. Therefore, the value of Epoch is very important for the evaluation of model performance. According to the experimental results, Epoch is set to 7. At this time, the analysis performance of the model is ideal.

### 3.3. Dropout Value Comparison Experimental Results

The introduction of Dropout can remove some neurons and update the weight and bias term through the remaining neurons in the process of forward calculation and back propagation. Then, the removed neurons are restored. Next, some neurons are removed again according to a certain probability, update the weight and bias term, and repeat this process until the end of neural network training. This can improve the generalization ability of the model to a certain extent and prevent the model from over-fitting. On the premise that other parameters remain unchanged, change the Dropout value. The accuracy results of the proposed model for the emotion analysis of microblog comment text are shown in Figure 6.

As can be seen from Figure 6, when the Dropout value is 0.3, the accuracy is the highest, up to 0.93. When the Dropout value is too low or too high, the accuracy performance is not high. This is because when the Dropout value is too low, too many neurons participate in training and are easy to fall into over-fitting. When the Dropout value is too high, too few neurons are left and easy to fall into under-fitting. Therefore, the Dropout value of the model proposed in the subsequent comparative experiment is set to 0.3.

### 3.4. Comparison of Training Results of Unidirection and Bidirection Long-Term and Short-Term Memory Models

The CNN-BiLSTM model is based on the combination of CNN and BiLSTM. On the one hand, because the convolution layer of CNN can effectively extract deeper and more abstract emotional features. On the other hand, the model combining the advantages of the two neural networks is better than the single neural network model. BiLSTM has a higher accuracy of emotion classification than unidirection LSTM because it can better take into account the previous and subsequent information. In order to intuitively show the advantages of CNN-BiLSTM model, compare it with the analysis results of CNN, LSTM, and BiLSTM models, and their accuracies are shown in Figure 7.

The experimental results of crawling Microblog data set show that BiLSTM can better analyze the information before and after the text, so as to improve the accuracy of emotion analysis. Compared with LSTM, its accuracy is improved by 2.89%. Similarly, the analysis accuracy of the BiLSTM model combined with CNN is higher than that of CNN-LSTM, about 0.935, which also demonstrates the feasibility of the proposed model.

### 3.5. Comparison with Other Algorithms

In order to demonstrate the performance of the proposed model, compare and analyze it with the models in references [13, 14] and [17], optimize the training parameters of each comparative experiment for many times, and select the experimental data with the best effect. The statistics of the experimental results are shown in Table 2.

As can be seen from Table 2, compared with other models, the analysis performance of the proposed model is the best, and its overall analysis accuracy is 0.94. Taking the analysis of positive emotion as an example, its analysis precision and recall are 0.95 and 0.89, respectively. Because the proposed model combines CNN and BiLSTM, it not only uses CNN to extract the deep features of the text, but also obtains the context information of the text based on BiLSTM, which is more conducive to the analysis of text emotion. Reference [13] implemented text emotion analysis based on dictionary model. Compared with deep learning algorithm, its analysis accuracy is low, lower than 0.80. Similarly, reference [14] used machine learning algorithm for text classification, which used automatic filtering to preprocess the text, but lacked comprehensive analysis and extraction of text features. Therefore, its accuracy is only 0.78. Reference [17] proposed a text emotion analysis method based on CNN, which can extract higher level sequences of text features through convolution layer, and the analysis accuracy is improved to 0.86. However, due to the lack of consideration of text context information, the overall accuracy of emotion analysis is reduced by 8.51% compared with the proposed model. Therefore, the effectiveness of the proposed CNN-BiLSTM model can be demonstrated.

## 4. Conclusion

The massive growth of data increases the complexity of the network environment. As a research hotspot of natural language processing, text emotion analysis has great research significance in public opinion analysis, user portrait, and recommendation system. Therefore, at this stage, with the continuous progress of artificial intelligence, it has important research value to realize effective emotion analysis through emotion calculation. Aiming at the problems of single word quantization and poor analysis accuracy in most of the existing deep learning algorithms in text processing, an emotion analysis model of microblog comment text based on deep learning is proposed. Because the output of LSTM hidden layer only depends on the output of the previous time, resulting in inaccurate analysis results, the proposed model combines BiLSTM and CNN to construct CNN-BiLSTM model. BiLSTM can obtain previous and subsequent information, and CNN can deeply mine text features. Thus, the accuracy of text emotion analysis is improved. Based on the crawled microblog data set, the experimental analysis of the proposed model shows that its overall accuracy is 0.94, which is better than other comparison models, and has a certain practical application value.

The proposed CNN-BiLSTM model includes a BiLSTM layer that can take into account the previous and subsequent information. Because the Gated Recurrent Unit (GRU) simplifies the gate structure in the LSTM, in the next research, it will consider using a bidirectional GRU network to replace the BiLSTM to improve the analysis efficiency of the model.

## Figures and Tables

**Figure 1:** Text emotion analysis model process based on deep learning.

**Figure 2:** Structures of CBOW model and Skip-gram model.

**Figure 3:** Structure of BiLSTM model.

**Figure 4:** Structure of CNN-BiLSTM model.

**Figure 5:** Comparison of training results under different Epochs.

**Figure 6:** Comparison results of Dropout values.

**Figure 7:** Comparison results of unidirectional and bidirectional LSTM models.

**Algorithm 1:** Pseudo code of Adamax optimization algorithm.

**Table 1:** Model parameter setting.

Parameter	Value
Sentence length	80
Batch size	128
Word vector dimension	300/330
Convolution window size	3,4,5
Number of convolution kernels	256
Number of BiLSTM hidden units	256
Activation function	ReLU
Loss function	Cross entropy
Learning rate	0.0001

**Table 2:** Experimental results of different models.

		Ref. [13]	Ref. [14]	Ref. [17]	Proposed model
Positive emotion	Precision	0.71	0.78	0.86	0.95
	Recall	0.83	0.84	0.82	0.89

Negative emotion	Precision	0.76	0.82	0.91	0.96
	Recall	0.69	0.75	0.80	0.88

Accuracy		0.74	0.78	0.86	0.94

## Data Availability

The data included in this paper are available without any restriction.

## References

[1] Braoudaki A., Kanellou E., Kozanitis C. (2020). Hybrid data driven and rule based sentiment analysis on Greek text. *Procedia Computer Science*.

[2] Hong S. K., Chong S. K. (2020). Analysis of IT service quality elements using text sentiment analysis. *Journal of Society of Korea Industrial and Systems Engineering*.

[3] Li W., Jin B., Quan Y. (2020). Review of research on text sentiment analysis based on deep learning. *Open Access Library Journal*.

[4] Chintalapudi N., Battineni G., Canio M. D., Sagaro G. G., Amenta F. (2021). Text mining with sentiment analysis on seafarers’ medical documents. *International Journal of Information Management*.

[5] Anandarajan M., Hill C., Nolan T. (2019). [Advances in analytics and data science] practical text analytics volume 2 (maximizing the value of text data) || sentiment analysis of movie reviews. *Using R*.

[6] Liao W., Zeng B., Yin X., Wei P. (2020). An improved aspect-category sentiment analysis model for text sentiment analysis based on RoBERTa. *Applied Intelligence*.

[7] Singh S. K., Sachan M. (2019). SentiVerb system: classification of social media text using sentiment analysis. *Multimedia Tools and Applications*.

[8] He H., Chen B. (2011). A smart sentiment analysis system in word, sentence and text level. *Advanced Engineering Forum*.

[9] Pang H. J. (2012). Text sentiment analysis-oriented commodity review detection. *Journal of Computer Applications*.

[10] Kirelli Y., Arslankaya S. (2020). Sentiment analysis of shared tweets on global warming on twitter with data mining methods: a case study on Turkish language. *Computational Intelligence and Neuroscience*.

[11] Li M., Xie L., Zhang A., Ren F. (2019). Reinforcement emotion-cognition system: a teaching words task. *Computational Intelligence and Neuroscience*.

[12] Nandwani P., Verma R. (2021). A review on sentiment analysis and emotion detection from text. *Social Network Analysis and Mining*.

[13] Ajitha P., Sivasangari A., Rajkumar R. I., Poonguzhali S. (2020). Design of text sentiment analysis tool using feature extraction based on fusing machine learning algorithms. *Journal of Intelligent and Fuzzy Systems*.

[14] Alqmase M., Al-Muhtaseb H., Rabaan H. (2021). Sports-fanaticism formalism for sentiment analysis in Arabic text. *Social Network Analysis and Mining*.

[15] Razzaq A., Asim M., Ali Z., Qadri S., Mumtaz I. (2019). Text sentiment analysis using frequency-based vigorous features. *China Communications*.

[16] Huang F., Zhang X., Zhao Z., Xu J., Li Z. (2019). Image-text sentiment analysis via deep multimodal attentive fusion. *Knowledge-Based Systems*.

[17] Xu F., Zhang X., Xin Z., Yang A. (2019). Investigation on the Chinese text sentiment analysis based on convolutional neural networks in deep learning. *Computers, Materials & Continua*.

[18] Lu X., Zhang H. (2021). Sentiment analysis method of network text based on improved AT-BiGRU model. *Scientific Programming*.

[19] Liu B. (2020). Text sentiment analysis based on CBOW model and deep learning in big data environment. *Journal of Ambient Intelligence and Humanized Computing*.

[20] Xu G., Yu Z., Yao H., Li F., Meng Y., Wu X. (2019). Chinese text sentiment analysis based on extended sentiment dictionary. *IEEE Access*.

[21] Al-Azani S., El-Alfy E. (2017). Using word embedding and ensemble learning for highly imbalanced data sentiment analysis in short Arabic text. *Procedia Computer Science*.

[22] Cheng Y., Yao L., Xiang G., Zhang G., Tang T., Zhong L. (2020). Text sentiment orientation analysis based on multi-channel CNN and bidirectional GRU with attention mechanism. *IEEE Access*.

[23] Kim Y., Kang M., Jeong S. R. (2018). Text mining and sentiment analysis for predicting box office success. *KSII Transactions on Internet and Information Systems*.

[24] Kotelnikov E. V. (2018). TextJSM: text sentiment analysis method. *Automatic Documentation and Mathematical Linguistics*.

[25] Zhang S., Wei Z., Wang Y., Liao T. (2018). Sentiment analysis of Chinese micro-blog text based on extended sentiment dictionary. *Future Generation Computer Systems: FGCS*.

[26] Zhou Q., Miao Q., Wang H., Xie W., Wang Y., Lu Z. Data science.

